The article "Mitochondrial Encephalomyopathy, Lactic Acidosis, and Stroke-Like Episodes (MELAS) in the 18th Century: Mitochondrial Disorders Are Not of Recent Origin" was published in 2022. Journal: Cureus.

# Mitochondrial Encephalomyopathy, Lactic Acidosis, and Stroke-Like Episodes (MELAS) in the 18th Century: Mitochondrial Disorders Are Not of Recent Origin

**DOI:** 10.7759/cureus.22314

**Published:** 2022-02-17

**Authors:** John Hayman, Steven Pavlakis, Josef Finsterer

**Affiliations:** 1 Clinical Pathology, The University of Melbourne, Melbourne, AUS; 2 Neurology, Downstate Health Sciences University, New York, USA; 3 Neurology, Krankenanstalt Rudolfstiftung, Vienna, AUT

**Keywords:** mitochondrial, seizures, stroke-like episode, mtdna, ocular hypertelorism, brachydactyly, cortical blindness, charles darwin’s illness, wedgwood illness, melas

## Abstract

Mitochondrial encephalomyopathy, lactic acidosis, and stroke-like episodes (MELAS) syndrome was one of the first mitochondrial disorders to be identified and characterized, being described as early as 1984. The clinical manifestations of MELAS vary but stroke-like episodes are a defining feature. Mutations in at least 17 mitochondrial DNA (mtDNA) located genes have been shown to be associated with this disorder.

Mary Ann, the youngest child of Josiah and Sarah Wedgwood, was born in August 1778 when Sarah was aged 44 years. Mary Ann was of short stature and was physically and mentally retarded. She suffered from partial and generalized seizures and episodes of cortical blindness. She died at the age of eight years. Descriptions of her illness remain and she is depicted with disabilities as can be seen in a family portrait. Her illness is consistent with MELAS. The illnesses of her elder siblings and of their mother are in keeping with a maternally inherited pathological mtDNA mutation, supporting this diagnosis.

Her illness is the key to the remarkable illnesses that affected the Wedgwood family. Through her eldest sibling, Susannah, married to Robert Darwin, the disorder was passed to the next generation, a generation that included Charles Darwin and his elder brother, Erasmus.

## Introduction

Josiah Wedgwood (Josiah I: 1730-1795), the famous potter, married a distant cousin, Sarah (‘Sally”) Wedgwood (1734-1815), and together they had eight children [1]. One child, Richard, died in infancy with sudden severe illness. Their last-born child, Mary Ann (1778-1786), died at a young age with a severe progressive illness. Her illness has been described in some detail in letters by Josiah to his friend and partner, Thomas Bentley (1731-1780). She is depicted with evidence of her disability in a portrait of the Wedgwood family by George Stubbs (1724-1806). Stubbs was famous for his portraits of horses and his attention to anatomical detail and anatomical detail is present in his portrait of the Wedgwood family. Mary Ann’s illness may be central to the understanding of the chronic illnesses that afflicted the Wedgwood and Darwin families, in particular Charles Darwin's illness.

The article "Mitochondrial Encephalomyopathy, Lactic Acidosis, and Stroke-Like Episodes (MELAS) in the 18th Century: Mitochondrial Disorders Are Not of Recent Origin" was published in 2022. Journal: Cureus.

## Case presentation

Mary Ann was the youngest child of Sarah and Josiah Wedgwood. From birth, she was noted to have delayed physical and mental development [1]. In the famous Wedgwood family portrait, painted by George Stubbs around 1780, she is shown as sitting in a small pull cart, an indication that she could not stand or walk (Figures 1, 2). In Stubbs' painting, she appears to have short fingers or brachydactylia - a condition that may occur with mitochondrial DNA (mtDNA) mutations [2]. The unusual shape of her dress may be due to padding, necessary because of absent bowel and bladder control. She had recurrent convulsions and at times was in status epileptics. These attacks were followed by periods of post-ictal paralysis and episodes of cortical or sub-cortical blindness, with increasing impairment.

**Figure 1:** The Wedgwood family, as painted by George Stubbs around 1780. The famous painting of the Wedgwood family, commenced c. 1780. From left to right: Mary Ann (seated in the pushcart), Sarah (standing beside her), Tom (on horseback), Catherine (pulling the cart), Susannah (later to be Charles Darwin's mother, on horseback), Josiah II, John (on horseback), and the parents, Sarah and Josiah (seated). Photocopied from [3]. Copyright: Wedgwood Museum/WWRD; used with kind permission.

**Figure 2:** Enlarged inset from Figure 1, showing Mary Ann seated in a cart, partly supported by her elder sister, Sarah. George Stubbs is famous for his attention to detail. Note Mary Ann's short fingers (brachydactylia) and the curved little finger (clinodactyly) seen on her right hand. The shape of her dress may result from padding necessary because of a lack of bladder and bowel control. Sarah, beside her, is shown with mild ocular hypertelorism. Photocopied from [3]. Copyright: Wedgwood Museum/WWRD; used with kind permission.

A letter from her father, Josiah Wedgwood, sent in November 1779 to his good friend, Thomas Bentley, is as follows: “Our little girl, Mary Ann, breeds her teeth very hardly, and unfortunately several of them are pushing forward at the same time. This brought on convulsions that lasted thirteen hours without intermission to the first attack, which was on Friday morning. And when this left her we found she had lost the use of her arm and leg on one side (postictal hemiplegia). She had a slight return (of fitting) for about half an hour the last night but is better again today” [3].

On the 23rd of November, Josiah wrote again: “… We thought our little girl much better yesterday. She is lively and playful, more so than we had observed since her illness, but this morning she is fallen off again and has had some return of spasms in her face. … When these convulsive remains leave her, we are not without hopes that the use of her limbs may be restored, though at present she does not attempt to make the least use of them, but makes use of her mouth in a hundred little instances to assist her other hand in the management of her playthings” [3].

The article "Mitochondrial Encephalomyopathy, Lactic Acidosis, and Stroke-Like Episodes (MELAS) in the 18th Century: Mitochondrial Disorders Are Not of Recent Origin" was published in 2022. Journal: Cureus.

Mary Ann was born in August 1778, so she would have been 15 months old when the episode occurred. No mention is made of the loss of sight in the first letter but in December 1779, Josiah reported: “Our dear little girl has got her sight again very perfectly we hope, & her limbs are recovering their wonted use every day. She is quite well & wild as a little buck, or rather a doe if you please” [3].

Unfortunately, her illness continued and worsened. A further letter, written in 1784, describes her inability to see (Figure 3). A transcription reads: “After writing to my dear friend yesterday evening I tried various methods to discover what degree of sight our poor child had left, and of what nature the defect might be. Before I went to Lichfield I conjectured that she had lost the faculty of adapting her organs of vision to the distances of objects, which would occasion a confused, and double vision, and I was the more confirmed in my conjecture from her seeming at first sight to (be) frightened at her nurse, or sister, or those of whom she was the most fond before, and Dr (Erasmus) Darwin to whom I mentioned these circumstances was of the same opinion. But when I could not make her perceive any object the last night ’till I touched her with it, I was very much alarmed for both her eyes…. I am not very well this morning though my fears are much less for my little girl this morning, as I find she can see by daylight, though not very distinctly, and I apprehend double from her sometimes putting her hand on one side of anything she offers to take at the first effort, when she tries again ’till she gets hold of it. I hope she will get the better of this defect, by practice, if her fits do not return, and I am exceedingly happy now to be assured that she has any sight at all remaining” [3].

**Figure 3:** A letter written by Josiah Wedgwood to his friend and partner, Thomas Bentley, around 1783. The transcript of this letter is in the above paragraph. The letter gives a striking account of cortical blindness as experienced by the little girl. Photocopied from [3]. Copyright: Wedgwood Museum/WWRD; used with kind permission.

Dr. Erasmus Darwin, Charles Darwin's grandfather, was a close friend of Joshua Wedgwood. He treated the little girl, and believing her convulsions were due to teething, incised her gums, placed her in a cold water bath, and administered electricity (galvanism). Not surprisingly, she failed to improve and suffered progressive physical and cognitive decline. She died at the age of eight.

The article "Mitochondrial Encephalomyopathy, Lactic Acidosis, and Stroke-Like Episodes (MELAS) in the 18th Century: Mitochondrial Disorders Are Not of Recent Origin" was published in 2022. Journal: Cureus.

## Discussion

Mary Ann's illness appears to have many of the clinical features of mitochondrial encephalomyopathy, lactic acidosis, and stroke-like episodes (MELAS), a syndrome that was first described in 1984 [4]. MELAS is one of the first diseases found to be due to pathological mtDNA mutations [5]. Mary Ann had short stature, intellectual disability, focal and generalized seizures, and stroke-like episodes, and from the description given by her father, she also had recurrent, transient cortical blindness. This description of her illness (1780s), written 200 years before MELAS was first identified, may be the first record of this disorder and the first record of a disorder due to a pathological mtDNA mutation.

Mitochondria produce most of the energy requirements for cells; cells vary in the actual numbers of mitochondria they contain, depending on these energy requirements [6]. Unlike other cell organelles, mitochondria contain their own DNA (mtDNA). MtDNA mutates more commonly than nuclear DNA; cells with mtDNA mutations frequently contain both wild type (normally functioning) mtDNA and mutant mtDNA, a condition referred to as heteroplasmy. Disorders due to pathological mtDNA mutations have symptoms that relate to the failure of energy production, rather than relating to the actual mtDNA mutation. When a cell divides, mitochondria flow randomly to daughter cells so that these may vary in their levels of heteroplasmy.

Illnesses due to mtDNA abnormality are maternally inherited as all mitochondria in the zygote are derived from the ovum. In developing ova, the number of mitochondria is initially reduced but then proliferates as development proceeds, resulting in a mature ovum that contains many thousands. As a result of this developmental "bottleneck," different ova from one mother may vary greatly in the number of normal and abnormal mitochondria that they may contain. This initial variation is compounded by normal and abnormal mitochondria passing randomly to daughter cells in the developing zygote. This initial varying level of heteroplasmy in different fetuses and subsequently in different tissues in the one fetus results in very variable symptoms and severity of illness in the progeny; progeny who have all inherited the same mitochondrial abnormality. Such variability is demonstrated in this family history.

Mutations in 17 different mtDNA genes are known to be associated with MELAS [7]. It is assumed that Mary Ann was born with one of these mutations, inherited from her mother, and, as will be shown, her siblings may have shared the same mutation but with lower levels of heteroplasmy.

The article "Mitochondrial Encephalomyopathy, Lactic Acidosis, and Stroke-Like Episodes (MELAS) in the 18th Century: Mitochondrial Disorders Are Not of Recent Origin" was published in 2022. Journal: Cureus.

Family history

Mary Ann’s older siblings also had illnesses, less diagnostic but nonetheless consistent with an inherited mitochondrial disorder. These have been described elsewhere [8]. Susannah (“Sukey,” 1765-1817), the eldest child, married Dr. Robert Darwin and was Charles Darwin’s mother. She had chronic, low-grade illness and famously complained: “everyone seems young but me.” She suffered from arthritis and like her mother before her, had hyperemesis with pregnancies. She died with probable peritonitis, possibly secondary to acute pancreatitis, a recognized occurrence in mitochondrial disease [9].

John (1766-1844), the eldest son, experienced tremor, “essential tremor,” all his life. The third child, Richard (“Dicky,” 1767-68), died suddenly at 10 months with an acute abdominal complaint. Josiah (Josiah II, 1769-1843) developed Parkinson’s disease in later life. Tom (1771-1805) suffered severe headaches and abdominal pain from childhood, dying at an early age with morphine overdose [10,11]. Catherine (“Kitty”) Wedgwood (1774-1823) was described as “somewhat masculine” and “the least attractive of the sisters” [12]. She was never married. In later life, she developed an abdominal tumor that reached an immense size. Her masculine appearance suggests that she may have had a pituitary adenoma or polycystic ovary syndrome, also known as Stein-Leventhal syndrome, the commonest cause of such endocrine effects in the female [13]. Polycystic ovaries are a recognized occurrence in association with mitochondrial disease [14]. Patients with this syndrome may develop cystic ovarian tumors [15], and these, as they were then untreated, may become very large.

Sarah (1776-1856) had no history of illness, but in the portrait of the family, she is depicted as having ocular hypertelorism (Figure 2), a condition described with mitochondrial mutation [16].

The mother of this generation, also named Sarah, although living to old age, was chronically unwell with arthritis and other symptoms [1]. The third generation, Susannah’s children, in particular Charles Darwin and his elder brother Erasmus, also had an illness. Charles’ illness, with numerous symptoms, has been described in detail elsewhere [8,17].

Except in various royal families, there would be few, if any, comprehensive family histories giving such detailed accounts of illness. The illnesses of many of the Darwin/Wedgwood family members are the type of illness that may have occurred in any large family at that age. Deaths in infancy were common. Although some of these illnesses are “strange” with vague, chronic symptoms and not readily diagnosed, they are not necessarily mitochondrial in origin. The argument for a mitochondrial link, however, becomes more compelling when the illnesses of Tom Wedgwood, who today would be diagnosed as having abdominal migraine, and that of the youngest sibling of the mother’s generation, Mary Ann, described here, are considered. The argument for a mitochondrial disorder is intensified again when these are joined with the descriptions of the chronic illnesses of Charles Darwin and his brother Erasmus (1804-1881). Their presentation, rather than signifying psychological illnesses, indicates probable mitochondrial disorders.

The article "Mitochondrial Encephalomyopathy, Lactic Acidosis, and Stroke-Like Episodes (MELAS) in the 18th Century: Mitochondrial Disorders Are Not of Recent Origin" was published in 2022. Journal: Cureus.

It is this illness of Mary Ann, an illness that seems typical of a severe childhood-onset mitochondrial disorder, that may be the key to the understanding of the chronic ailments affecting the Wedgwood and Darwin families, in particular, the debilitating illness that afflicted Charles Darwin.

## Conclusions

The detailed description of the illness and the depiction of Mary Ann Wedgwood, born some 240 years ago, allow for a credible diagnosis of MELAS; an illness that occurred 200 years before the clinical identification of the syndrome.

It may be assumed that if this illness was due to a pathological mtDNA mutation, then other members of the Wedgwood family and their matrilineal Wedgwood/Darwin descendants carried the same mutation with varying levels of heteroplasmy.

The unusual, chronic illnesses that afflicted members of the Wedgwood and Darwin families may be explained by the sharing of an inherited pathological mtDNA mutation of the MELAS type, with differing phenotypic manifestations. Charles Darwin's illness may be explained by his inheritance of this same mtDNA mutation.
